This article has been retracted.

# Analysis and Practice of Applying Oriented Teaching Method to Improve the Effect of College English Teaching

**DOI:** 10.1155/2022/9689181

**Published:** 2022-05-28

**Authors:** Hua Yang

**Affiliations:** College of Foreign Studies, Guilin University of Electronic Technology, Guilin 541004, Guangxi, China

## Abstract

The Ministry of Education of my country released the first “national standard” in January 2018, clearly stating that it is necessary to attach importance to and improve the ability of undergraduates. Through the analysis of the research results in this field at home and abroad, this study finds that the thinking ability training strategies that can be provided in the previous research are relatively scattered, and there is a lack of effective training methods and guidance. Therefore, Dr. Wen Qiufang proposed the teaching method of “production-oriented approach.” “Production-oriented approach” includes driving, promoting, and re-evaluation, in which the training content is integrated into each link. Therefore, this study combines training and Production-oriented Approach, and using this theoretical basis in the English teaching classroom can explore better. It provides a new way for the cultivation of college students' English thinking ability. In the actual classroom teaching, the production-oriented teaching method is used to teach English to the students during the research process. After the teaching course is over, the teaching data are collected and analyzed with SPSS 25.0 software, and the data results are displayed. It can be seen that applying the Production-oriented approach to English classroom teaching can indeed improve the level of domestic college English students and provide a reference approach and method for students' English training, and this method is effective and feasible.

## 1. Introduction

### 1.1. Research Background

In recent years, Western developed countries have begun to pay attention to how to improve learners' ability. After years of research, its ideas, methods, and system theory have been relatively perfect. Due to the implementation of exam-oriented education in China, we pay attention to students' examination results and despise the cultivation of students' quality. In particular, the cultivation of ability is very lacking. In recent years, the cultivation of ability has gradually been valued by everyone. How to cultivate students' ability, many researchers have always believed that “skills should be integrated into specific research projects, or combined into specific contents, rather than being taught as an independent discipline” [1–4]. In English writing, it includes knowledge links such as reasoning, proof, evaluation, and logic, which need to be fully thought and related to the content. On the other hand, we also need to think in the writing process, from the overall planning and layout of the article to the correct value judgment, logical reasoning, and other links. Therefore, we need the ability of examining ability and critical thinking when writing [5]. So, writing is a good way to train learners' ability.

Production-oriented Approach is to use challenging and social dynamic scenes to fully mobilize students' enthusiasm and interest in learning and create students' psychological motivation for English writing. This output-oriented method is guided by the teaching goal. In teaching, it starts with “expression,” selectively selects words, combines “learning” and “use” in teaching practice, and sublimates the whole teaching process by evaluating the steps of “learning.” Learners learn in “use” and evaluate in “learning.” Finally, let the students “express” in the form of an article. Applying this method to English teaching can not only improve learners' writing level, but also exercise learners' English ability. At the same time, it can also solve the “separation of learning and application” in the current education system.

This study attempts to explore the use of output-oriented teaching method to carry out teaching, so as to verify the impact of this method on the ability training of non-English majors. The main research contents are as follows:

1. Research content and focus. In this study, the training of English thinking ability is closely combined with the output-oriented method, and the practice is carried out based on the writing teaching, which overcomes the defects of no systematic teaching methods in the previous academic circles when discussing the training strategies of thinking ability, and provides some reference for the training of thinking ability.
2. Research methods focus. Taking the English classroom teaching of college English as the experimental site, this study innovates the English classroom teaching methods through the output-oriented teaching method, analyzes how the students' use the learned knowledge to complete English writing in the new teaching mode, solves the problems, and finds their own shortcomings, so as to improve the students' English practical thinking ability..

### 1.2. Research Purpose

Cultivating learners' ability is the common choice and requirement of many well-known universities in the world. China also clearly requires colleges and universities to cultivate students' learning ability. However, at present, there is still a lack of ability training in the domestic college classroom, which is still based on skill training. From the perspective of domestic educational development in the future, the training of ability is bound to be paid more and more attention by educators. Therefore, many experts are also conducting deeper theoretical research and making innovations in curriculum compilation, teaching methods, and so on. Based on the research of experts, this study adopts the POA method to carry out writing courses and looks for ways to implement training to help learners improve their ability.

### 1.3. Research Significance

In recent years, although it has been widely recognized in the field of English teaching in China that English is of great significance in training students' thinking ability, the research in this field is far from enough. Some researchers have analyzed the characteristics and prominent problems of students' thinking ability and pointed out that the content of students' English writing is empty and lack of logic. However, in the process of English education in the past, few people have studied effective ways to solve this problem. In view of this, how to reasonably infiltrate the training of thinking ability in the process of English education in order to improve learners' thinking ability has become the focus of common concern in today's English education.

After sorting out relevant materials and observing some teachers' classroom teaching, we can see that many teachers lack the guidance of specific ideas in classroom teaching, which leads to the disconnection between teachers' classroom teaching and students' awareness education. Therefore, this study will start from English teaching, adopt the new ability theory model, and explore the ways of cultivating non-English majors' ability based on the theoretical system of output-oriented method. Through the practical methods put forward by the teachers in the classroom, we can change the situation of emphasizing language ability and less thinking ability in the traditional teaching of the school, so as to realize the all-round development of college students' overall literacy.

## 2. Theoretical Basis of the Study

### 2.1. Capability Theory and Related Models

#### 2.1.1. Evolution and Definition of Capability

The source of critical thinking comes from Socrates' questioning method. Socratic questioning usually needs to test or question the premise or hypothesis of logical structure [6, 7]. John Dewey is the father of modern critical thinking. He defined critical thinking as “a hypothetical form of knowledge that trusts or encourages trust, and it tends to make some results and give them active, persistent, and prudent consideration” [8]. His definition emphasizes the importance of understanding facts and evaluation to people as well as the expression of faith by reflection. Some researchers label it as the definition of “critical thinking,” Dewey et al. call it “reflective thinking,” [9] and Bloom et al. think it is “wisdom and skill” [10]. It is also an appropriate way of thinking and criticizing the truth of things. Wen advocates redefining the thinking ability on the basis of previous research, that is using the correct method, carrying out conscious thinking, and making reasonable conclusions [11]. She also pointed out that human thinking ability is mainly composed of two levels: thinking tendency and skills [12]. This thesis will carry out scientific research and practice according to this concept, mainly focusing on non-English majors in domestic colleges and universities, and explore ways of ability training.

#### 2.1.2. Capability Model and Theory

Facione put forward the theory of two-dimensional structure in 1990, pointing out that human ability is composed of thinking tendency and cognitive skills [13]. Thinking tendency refers to the thinker's own critical thinking, and cognitive skills refer to the ability to focus on intelligence in the process of thinking. Capable thinkers not only have the ability to think about problems, they will also apply the ability of thinking to critical problems. Thinking tendency and cognitive skills play an important role and influence on the development of personal ability. They complement each other and are indispensable.

The theoretical knowledge framework mainly covers seven aspects: exploring truth, thinking openness, analytical method and logical reasoning, systematic ability, self-confidence, thirst for knowledge ability, and psychological maturity, of which

1. Seeking the truth refers to the objective and true state of mind when seeking the facts or seeking the truth. It shows that even when the conclusion pursued by an individual conflicts with his own will and values, he can reflect on himself and improve.
2. Openness of thinking refers to the degree of openness in personal thinking, that is the degree of recognition of the correctness and correctness of one's own views, and also includes the degree of acceptance of one's views in various own views.
3. The analytical method and logical reasoning refers to the degree of individual recognition of problems in their own and others' views, that is individuals can use evidence to solve problems and predict possible results.
4. Systematic ability refers to the ability to put forward plans and problems clearly and systematically.
5. Self-confidence refers to having confidence and interest in their own data analysis ability, reasoning, and demonstration process and conclusions and being able to raise their own questions and put forward reasonable opinions.
6. Interest and thirst for knowledge refers to showing strong interest in complex and unknown problems, being willing to explore their causes and methods, and paying attention to mastering and understanding, so as to make continuous progress.
7. Maturity means being extra cautious in making judgments and being able to make an expedient judgment with an objective and correct attitude according to various handling methods.

### 2.2. Definition and Content of the Theoretical System of “Production-Oriented Approach”

In China's exam-oriented education mode, there is always a situation of “separation of learning and application.” In order to solve this problem, the Production-oriented Approach has been developed. The advantage of POA is that it closely combines teaching materials with teaching methods in students' learning and is in a leading position. This Law consists of the following parts:

The first part is “teaching theory”: it is the theoretical basis of POA, which plans the overall framework, teaching objectives, and teaching direction of classroom teaching. The second part is “classroom practice”: in classroom teaching, every link of the content of classroom activities is checked and solutions are put forward according to the problems. The third part “teaching procedure”: it is the main means and process to achieve the educational goal of output-oriented method. It is the main carrier to test the process of “classroom practice” and implementing “teaching theory” [14].  Figure 1 clearly illustrates the structure and correlation of various elements of the basic theoretical framework of the output guidance method.

The three stages of POA (production-oriented approach) classroom teaching are driving, facilitating, and evaluation. In each teaching stage, teachers play a guiding role. From the results of the experiment, the three stages are interconnected and cooperate with each other, and there are many small links in the three stages. In each classroom teaching, the small links in each stage are constantly cooperating with each other and playing a role [15].

First of all, in the driving stage, it uses “output-input” to replace the traditional classroom teaching sequence of “input first and then output” to induce learners to find existing problems, find their own defects, and trigger autonomous learning interest and potential motivation. This is an important process for learners to use their own strength to realize autonomous thinking, which is completely different from the traditional teaching method, and to focus on cultivating students' strengths in all aspects. Applying the overall theoretical framework of output-oriented method to English classroom teaching can guide students to use their ability to achieve teaching objectives, which can be used as a reference for integrating ability into classroom teaching and becoming a teaching method in the future.

## 3. Research Design

According to the phenomenon of “absenteeism” commonly existing among college students pointed out by Dr. Huang Yuanshen, combined with the provisions of the latest national standard on the cultivation of college students' ideological core quality and the attention paid to the cultivation of students' thinking ability, the content of this article aims to explore the strategies and ways of cultivating students' thinking ability by using the output lead-in teaching method. Specific research issues include

1. What is the capability status of English majors in colleges and universities all over the country?
2. What is the impact of English writing education based on output-oriented approach on cultivating students' ability?
3. What are the specific contents of English majors' ability training strategies?

### 3.1. Research Object

The research object of this study is the non-English major students of a normal university in Guangxi. In the sophomore middle school, there are 178 students in four classes, including 28 boys and 150 girls. The students of this major are about to face the beginning of the CET-4 test, and the English score accounts for 20% of their total test score. This research method will help students improve their academic performance, so both teachers and students cooperate with this experiment very much. After comparing the average score performance of each class, they think that the difference between the sum of the average score of class 1 and class 3 and the sum of the average score of class 2 and class 4 is small, so they decide that class 1 and class 3 are the experimental classes and take class 2 and the class 4 as the control classes.

### 3.2. Research Tools

The project adopts a combination of quantitative data analysis and qualitative scientific research. The survey process is divided into questionnaire and specific interview. After getting the conclusion, SPSS 25.0 is used for data analysis.

#### 3.2.1. CTDI-CV Scale

In this scientific research, the author used (CTDI-CV) to complete the per and posttest of scientific research. CTDI was designed in 1992. It is one of the tools used to analyze the seven aspects of learners' thinking ability. The specific contents of the seven aspects are: systematization, analysis, openness of thinking, seeking truth, self-confidence, knowledge maturity, and thirst for knowledge. Professor Peng MEICI revised it according to the domestic cultural habits to be more suitable for Chinese learners. Professor Peng added 10 items to each of the seven aspects in the original orientation table, and each item has six standard levels, ranging from “very agree” to “very opposed.” Students choose the corresponding level content according to their own feelings, so as to express their actual feelings. In the option of thinking ability, the score is between 10 and 60. Among them, 40 is the dividing score between positive thinking and negative thinking. For example, if a student's score in a certain aspect exceeds 40, the student's thinking ability in this aspect is positive. If it is lower than 40, the student's thinking ability in this aspect is negative. In the overall evaluation, students' scores are about 70–420. If the student's test score is less than 210, it indicates that the student has poor ability in the overall classroom teaching. If the student's test score is between 210 and 280, it indicates that the student's thinking is in a contradictory state in the classroom teaching. If the student's test score is more than 280, it means that the student's thinking is positive in classroom teaching. When the student's test score is more than 350, it means that the student's ability is very good. The details are shown in Table 1.

In order to more truly reflect the actual learning situation of students, this test selects the items in the table according to the actual situation of students. Finally, five options suitable for the actual situation of students are selected in each level. After analysis with SPSS software, we can get validate the analysis as shown in Table 2.

It can be seen from the above table that if the KMO value is less than 0.820 or greater than 0.8, it indicates that the data have certain effectiveness and have strong effectiveness. In order to facilitate the statistics and data calculation and analysis, the score range of the original questionnaire is converted in the same proportion, and the following table is determined to prevail (Table 3).

In order to more specifically grasp the students' ability, the students' actual acceptance of this teaching method, and the problems they face and encounter, this study randomly selected 12 students in the experimental class to conduct a semistructured interview. There are 10 multiple-choice questions in the interview outline, which roughly covers about the obstacles and problems faced by students in the learning process and the understanding of how to cultivate students' thinking ability and the changes in teaching.

### 3.3. Research Process

#### 3.3.1. Pretest of Capability Level

This study is planned to be conducted in the second semester of the 2020–2021 academic year in the sophomore year of an English major in a domestic university for 8 weeks. Before the research, the researchers conducted a pretest on all students in the class to obtain and analyze the relevant data of the ability level and writing level of the research object and used SPSS 25.0 after an independent sample *t*-test was conducted on the data of the experimental class and the control class to test whether the level is sufficient. At the same time, the revised thinking tendency questionnaire is also used to study and pretest the level of thinking ability of the respondents. After the collection and testing of this test questionnaire, it is proved that it is a valid answer sheet, with a total of more than 178 copies. When using SPSS 25.0 after the independent sample *t*-test with software, it is found that there is no significant difference in the ability level between the two classes (see Tables 4 and 5), which basically meets the needs of writing teaching experiment.

#### 3.3.2. Using the Output-Oriented Teaching Method to Carry Out Teaching Experiment

While starting the experiment, in the experimental class, the teacher will use the output-oriented method to carry out teaching, whereas in the control class, the traditional English mode will be used to carry out teaching, so as to facilitate comparison and analysis in the future. After discussion with the teacher, the author decided that the main content of the subject is to select appropriate target materials from teaching materials or auxiliary materials, which can be ecological environment, physical health, classroom ideas, etc., and the specific process is as follows: (as shown in Figure 2).

The first link: data-driven link. The teacher asked the students to preview the content of this class before starting and find relevant materials in the pro-phase. In class, the teacher uses multimedia equipment to let the students watch videos related to the topic. Thereafter, the teacher asks the students in detail about their impressions and feelings and asks the students to discuss the specific content and views and so on of the video in groups. In this link, the teacher induced the students' interest by establishing the actual scene, mobilized the students' enthusiasm, understood the lack of their own knowledge, improved the teaching effect, and laid a good foundation for the smooth development of classroom teaching in the later stage.

The second link: teaching facilitation. The teacher guides the students to learn the content of this class through the prepared materials, so that the students can clearly understand their writing objectives and plan and know how to express them smoothly. In the process of writing “output,” teachers are leaders and promoters, and they timely answer and deal with the difficulties and questions of students in the process of “output,” actively guide students to participate in teaching activities, and unite and cooperate to achieve the goal of “output” of students. In this link, students need to do the following work:

The first is preparation, including viewpoint, argument, or logical reasoning. Second, for the preparation of discourse factors, the teacher must also let the students prepare the words, phrases, or sentences related to the topic. Enable each student to choose various materials related to self-writing output.

Finally, the preparation in the field of thinking logic is often related to the pattern of the overall article content and the correlation between various fragments, which requires teachers' guidance.

The per class preparation link can enable the teacher to play a guiding role, help each student understand the relationship between thinking ability training and reading language ability training, and also enable each student to carry out thinking preparation, reading language preparation, and thinking logic preparation at the same time, so as to output the results of thinking in the form of writing in different languages.

Evaluation link. Including students' self-evaluation, network sharing, and teachers' comments. In the operation of each student's self-evaluation, the teacher should guide the students to find their own problems, such as grammatical errors and spelling errors found in the process, and actively correct them.

Mutual evaluation link. In this link, students check each other's ideas and say their own ideas. While discovering classmates' problems, they also find their own shortcomings, so as to correct and supplement their own mistakes and deficiencies.

In teacher evaluation link, teachers give effective feedback to learners' writing output, mostly in the form of encouraging language, and help learners correct some mistakes. The key is to help learners rebuild self-confidence, so as to make future teaching and practice more smoothly.

#### 3.3.3. Post-Test of Capability Level

At the end of the experimental period, this study used CTDI-CV scale to carry out the ability post-test, using SPSS 25.0. This study makes a systematic data analysis on the test data of the prrtest and post-test. This study uses the method of random sampling and selects more than ten students to carry out semistructured interviews in order to understand the students' emotional attitude and acceptance of the new teaching methods and puts forward some reference suggestions for teachers' future education.

## 4. Experimental Analysis

This study makes statistical analysis and explanation on the experimental data obtained from this research, and uses SPSS 25.0 software system for data analysis. The specific contents include: first, the thinking ability and pretest results of the research object are statistically analyzed in order to master the thinking ability and current level of the research object. Then, the pretest and post-test results between the experimental class and the control class are used by SPSS 25.0 software system in which independent sample t-test was carried out and its differences were analyzed, so as to explore the impact of using output-oriented teaching method to carry out education on students' ability level.

### 4.1. Comparison and Analysis of Pretest Results between the Two Groups

At the beginning of the experiment, CTDI-CV measurement table was used to investigate all sophomores of non-English majors (including experimental class and control class). The pretest data of students' level were obtained, and the data were analyzed and studied. Therefore, the level of the two groups of students was understood, and SPSS 25.0 was used to conduct independent sample *t*-test on the data of the experimental class and the control class. In-depth analysis of the level of the two teams and the test results are shown in the table below:

First, the *T*-test results of independent samples are evaluated as a whole.

According to the above, by analyzing the test of single sample *t* in the pretest results, the following results can be obtained, SIG average values are greater than 0.05 (0.519 > 0.05), if there is - sig. If it exists, it is the result based on the assumption that the variance is the same. If the value on both sides is 0.214 (0.214 > 0.05), it indicates that there is no obvious difference in thinking ability and level between the experimental group and the control group, and it also indicates that the overall thinking level of the two groups is basically at the same level (as shown in Tables 4 and 5).

The test conclusion of single sample *t* can also be reflected by the comprehensive analysis and evaluation results of relevant pretest questionnaires of the test group and the control group (Table 6).

As shown in Table 6, the average values of the experimental group at different levels are: seeking truth: 20.98, open thinking: 20.18, analytical reasoning: 21.16, systematic ability: 20.79, self-confidence: 19.71, thirst for knowledge: 19.48, and maturity: 20.14. The order of mean scores from high to low is: analytical reasoning > seeking truth > systematic ability > open thinking > maturity > self-confidence > thirst for knowledge. The higher the score, the better the learner's performance in this area. Analytical reasoning ability is the most outstanding project content among the seven experimental contents of thinking and learning ability. Relatively general performance is seen in the ability to seek truth, systematic ability and open thinking. Maturity is average in the seven projects, while the projects with relatively poor performance and contradictory performance level are self-confidence and thirst for knowledge.

The average values of the control group at different levels are: seeking truth: 20.34, open thinking: 19.29, analytical reasoning ability: 21.06, systematic ability: 19.93, self-confidence: 19.51, thirst for knowledge: 18.75, and maturity: 20.19. The average scores of the students in the control class at all levels from high to low are: analytical reasoning > seeking truth > maturity > systematic ability > self-confidence > open thinking > thirst for knowledge. It can be seen from the above table that the students in the control class perform best in seven aspects: analytical reasoning, seeking truth, and maturity for relatively good performance; systematic ability, self-confidence, and open thinking for relatively general performance; and thirst for knowledge for relatively poor performance. However, different from the experimental class, the control class has reached a relatively positive level only in the three dimensions of analytical reasoning, seeking truth, and maturity, while the rest have reached a contradictory level.

This study not only makes different levels of mean statistics on the students of the two classes, but also makes an independent sample *t*-test on the pretest data of the two classes to compare their different force levels. It can be seen from Table 6 that the *P* value in each sub-plan of the experimental class and the control class is greater than 0.05, which shows that the ability difference between the two classes of students in the project is not obvious, that is the ability level of the two research objects is not different, and they all meet the experimental conditions.

However, according to the level evaluation criteria of the adapted version introduced above, we can see that the average score of each subject in the control class and the experimental class is 21.16 and 21.06 in analytical reasoning subject; in addition to the analytical reasoning, the scores of the two classes are slightly more than 20 in the level of seeking truth and maturity, while in the two dimensions of open-minded and systematic level, the score of the experimental class is higher than 20, which is at a positive level. In other subjects, the ability level of the two classes is about 15–20 points, which belongs to the contradictory level. It can be seen that the training task of students' English thinking ability is very urgent and arduous.

### 4.2. Comparative Analysis of Post-Test Results between the Two Groups

Before the end of the new semester, this experiment carried out the pretest and post-test of thinking ability in the experimental class and the control class again, and used SPSS 25.0 to complete the analysis.

The first is the overall evaluation of the independent sample *t*-test conclusion.

As shown in Table 8, in the independent sample *t*-test results of the two groups, SIG. The absolute values of are equal to 0.05 (0.845 > 0.05). Therefore, it is correct to assume that the variances are equal Sig. The average value of both sides is 0.022 (0.022 < 0.05), indicating that in the post-test of capability level, the talent level between the control group and the test group shows obvious differences, that is their overall talent level is very different (see Tables 7 and 8). According to the analytical evaluation of the ability level post-test of the experimental group and the control group, the conclusions of the independent sample *t*-test are as follows.

As shown in Table 9, in the seven items of thinking ability post-test, the average number of the experimental class is better than that of the control group. Especially in the three dimensions of openness, analytical reasoning, and maturity, the average difference between the experimental class and the control class is 2.6 points, 3.5, points and 2.61 points, respectively. Moreover, the average scores of the students in the experimental class in all aspects have exceeded 20 points, indicating that the students' thinking ability has reached a positive level, while in terms of systematic ability, the scores of the students in the experimental class have exceeded 25 points, reaching a strong level. Moreover, the average score of the experimental class is 14.44 points higher than that of the control group, and the score difference is very obvious.

Comparing the pretest results of thinking ability, it can be found that although the average score of the experimental research class is higher than that of the control group, there is little difference between them, and the score gap in different dimensions is also very small. However, in the post-test, the post-test conclusion of the experimental class is more prominent than the pretest conclusion, especially in the three dimensions of open thinking, analytical judgment ability, and systematic knowledge. Compared with the pretest conclusion of the experimental class, its score has increased by 3.31 points, 3.8 points and 4.24 points, respectively, and its average score has also increased by 17.06 points compared with the pretest conclusion.

On the contrary, the score measured by the control group increased significantly in the dimension of systematic ability, with an average score of 3.21 points. However, in addition, the score of other dimensions did not increase significantly, and even in the dimension of maturity, the score also decreased significantly. In terms of total score, the overall score is only 5.995 higher than the pretest score of ability, but the effect is not outstanding.

The independent sample *t*-test was used to test the differences in seven aspects between the students in the practice class and the control class. The data results show that each data sample shows distinctive characteristics in seven aspects (*P* < 0.05), that is to say, there are differences in seven aspects of each data sample.

In addition, from all dimensions, the average score of the experimental class is significantly higher than the total average of the control class. At the same time, the average score of the total score of the thinking ability test of the experimental class is 159.51, which is also significantly higher than the total average score of the control class by 145.07, indicating that after using the output-oriented method to carry out the thinking ability and teaching experiment, the students' thinking ability level of the experimental class is significantly higher than that of the control class. It also proves that bringing the output-oriented teaching method into the teaching experiment is of great significance to the improvement in students' thinking ability.

### 4.3. Interview Results

After the completion of the teaching experiment, we immediately selected ten research objects in the experimental class, conducted an interview with the teaching outline, and recorded and analyzed the interview content. The interview conclusions include the following.

Question 1: eight students thought that there were problems at the beginning of teaching because the new teaching method had higher requirements for students' word quantity and cognitive reserve, so it was difficult to keep up with the teacher's rhythm at the beginning, but the new teaching method made them have a sense of participation, enthusiasm, and quickly adapt to the teaching method and rhythm.

Question 2: five students think they are most interested in task-driven links, because this link can help students expand their ideas, brainstorm, and arouse their thirst for knowledge. Two students believed that the facilitation link could help students master more social background and vocabulary involved in the topic and also understand how the teacher writes related topics. The rest of the students think that the comment link is the most rewarding, because after self-assessment network sharing content and teachers' comments, the students have a more sufficient understanding of their own abilities and the place of prone to mistakes, so they will be more serious and rigorous in their next writing.

Question 3: in terms of the improvement in thinking ability, each student affirmed that after the teaching class, they learn to look at problems from multiple perspectives, and their thinking problems will be more comprehensive. Some students find that their knowledge reserve is too small and their word reserve is too small, which limits their thinking ability and writing level. Some students believe that they will use their ability more actively in the process, and feel that it will play a very positive role in improving their writing level.

Question 4: students with low achievement say that there are indeed obstacles when using their ability to complete. It mainly comes from two factors, namely the lack of vocabulary and narrow understanding. Because of the lack of vocabulary, students are often unable to express their thinking ability smoothly in the process of writing. Sometimes, the use of thinking ability will make the creation unable to proceed smoothly because of the unfamiliar topic of creation.

For the last question, about the review of this semester, the students think that they have made great progress in English writing. The new teaching mode has increased their interest in learning keen on the materials and vocabulary related to the writing theme. Group discussion has broadened the students' thinking, and self-assessment and network sharing have enabled the students to have a clearer understanding of their own level.

Through the conclusion of the interview, we can see that the respondents are very positive about the teaching methods adopted in the teaching experiment, pointing out that this method is novel and fun, which can mobilize students' learning enthusiasm. At the same time, it can make students consciously use their thinking power to think and solve problems, and further find the differences between themselves and others in teaching, developing strengths, and avoiding weaknesses in order to improve learning.

## 5. Strategy Analysis

### 5.1. Driving Link

#### 5.1.1. Scene Settings

Scenario setting is the first step of the driving link. In the process, teachers must provide materials related to the topics of this writing course and provide students with all aspects that may be involved in the topics at the beginning of the course, such as economy and society, politics, literature, military, social history, academic issues, life, etc. The display methods can be divided into video, photos, music, etc. This material should not only fit the topic but also take into account students' interests and preferences or campus life experience. When the article is presented, teachers often have to create a relevant situation for students to participate in.

#### 5.1.2. Task Settings

After setting the scene, the teacher must set the output task. This is mainly reflected in the teaching plan. The plan must include all aspects of content and form. Teachers can also divide the course tasks into several small tasks to carry out teaching activities. According to the needs, the teaching content is divided into the following aspects: words, phrases, sentence patterns, articles, opinions, etc. Starting from the most basic vocabulary, learners can continuously improve their self-identity to English learns with the help of small tasks and then enhance their self-confidence.

### 5.2. Facilitating Links

In the output-oriented teaching method, the most important link is the facilitation link. In facilitation link, the focus of the teaching task is “output.” In the classroom, “output” teaching materials promote students' thinking, let students complete the teaching objectives from multiple angles, and improve their level through the teaching objectives they want to achieve. After a deep understanding of the content of the teaching materials, the teaching objectives can be achieved, and the “output” requires a clear point of view of the teaching materials, an appropriate organization of teachers' guiding language, and a reasonable teaching structure.

#### 5.2.1. Clear Positions

The last step of the output-oriented method is to let students clarify their own views and make statements based on them. When guiding students to form their own views, we can inspire students' multilevel thinking dimensions according to auxiliary materials, so as to clarify their own views. For example, the teacher can guide the students to think by asking questions, and then give the students six sentences, each of which represents a different perspective of thinking. After reading carefully, the students can clarify the arguments behind the sentences and summarize the relevance of the sentences, so as to establish their own views. Then the teacher issued the materials of the teaching objectives, and the students began to study the content, argument angle, and expression of the materials. Thereafter, the students began to divide into discussion groups to discuss their ideas and footholds on this material with their own team members. Finally, the students report in the group and share the information and views of the whole class on the Internet, and then the teacher will comment in detail.

#### 5.2.2. Guide Express in Language

After passing the previous link, the students have a certain understanding of the content of the writing materials. Then choose the important language items in the text as the practice goal and design and process them into different degrees of language training. Translation training can be designed according to the important sentences in the text. In translation, paying attention to the use of context and completing binding of training materials and training results facilitate future review and use and increase the sensitivity and proficiency of words and sentences.

#### 5.2.3. Understand the Logic and Write Output

In this link, teachers can first carry out the pretest work, that is, let students write the first article, and then the teacher read and appraise the article to find the problems caused by the pretest. Then, the teacher will launch a special introduction to help students understand the logical relationship between paragraphs from learning and use, and then write good fragments. Then, the teacher should also introduce the model text to the students and appreciate it together. Thesis appreciation can closely integrate reading and writing, which is a good teaching way. Specifically, students should first look at the whole article, then judge the composition of the article, and judge the relationship between “establishment” and “refutation.” Then, let the students look for ideas and arguments first, and finally give the basic structure of the paper. Through these links, students can have a clear understanding of the basic idea and structure of the paper, in order to provide reference for the basic structure of the paper to be written. After the above processes, they found their own defects, had their own opinions on the topic, and learned how to use sentences to express them. At the same time, through topic introduction and thesis appreciation, the students also had a relatively clear understanding of the composition logic of the works. Then, the teacher must guide them to complete the output exercises, that is giving them 45 minutes to complete and polish their works and check the learning effect [16−20].

### 5.3. Evaluation Link

This part is the last part of the “production-oriented approach” classroom teaching, including three sub-links: students' self-evaluation, mutual evaluation among students and teachers' comments, and teacher evaluation. Through accurate and reasonable evaluation and feedback, students can be encouraged to review and reflect on the teaching process again, so as to enhance their learning motivation.

In the students' self-assessment, students first check their opinions and contents repeatedly, focusing on the spelling, grammatical combination, and content structure of words. The key content of this link is to let students carry out inspection and thinking.

Then there is mutual evaluation among students. The students are divided into groups to check each other's article content, comment, and check the students' article content. In this link, the students can have a deeper understanding of the data and have a clearer understanding of the overall structure, logical level, language structure, and other aspects of their articles.

The last is teacher evaluation. In the evaluation link, teachers need to pay timely attention to whether students reflect reflective emotional characteristics in the process of writing learning, such as open-minded, self-confidence, strong thirst for knowledge, and other emotional characteristics. At the same time, teachers should also affirm the emotional characteristics of this active tendency formed by students in a timely manner, provide students with relaxed democratic learning atmosphere, and guide students to make objective and active emotional reflection and thinking. These can guide students to actively carry out cooperative practice, help students establish writing confidence, and then play a good effect of training thinking ability.

## 6. Conclusion

This study adopts the production-oriented teaching approach to carry out the English teaching experiment. After completing the comparative study of empirical data and pretest and post-test results, this study puts forward the following conclusions. The average score of pretest thinking ability of English majors in general colleges and universities is 142.45 points in the practice class and 139.08 points in the control school. Although the gap between the two is not big, and some scores are at contradictory levels, in the seven levels of thinking ability, the students in these two classes showed a relatively active level of analytical and reasoning activities, while the weak ones were self-confidence and intellectual curiosity.

In the classroom teaching experiment, there was no significant difference in the average ability of the experimental class and the control group. However, after the writing teaching experiment, the post-test results of the ability of the experimental class and the control group showed that the total average score and the improvement degree of the experimental class were higher than those of the control group. Therefore, the development of output-oriented teaching method is of great significance to the improvement in college students' professional English teaching level.

In the driving link, teachers must first set the topic situation, so that students can be in it, and in the promotion link, teachers must also be divided into several parts. These sections help students understand the logical relationship between the composition of the essay and the ideas of the essay. The last link is the student evaluation link, which can objectively and comprehensively reflect the shortcomings of the students so that the students can clearly and directly find the shortcomings of the article comments, and check the content of the students' articles, which is conducive to the students' self-examination, enhance their strengths and avoid weaknesses, and check and fill in the gaps.

## Figures and Tables

**Figure 1:** POA theoretical system diagram.

**Figure 2:** Writing teaching process guided by output-oriented method.

**Table 1:** CTDI-CV rating criteria.

Gauge	Subitem score	Overall score
Negative level	<30	<210
Contradiction level	30–40	210–280
Positive level	40–50	280–350
Intensity level	>50	>350

**Table 2:** Validity analysis of adapted CTDI-CV questionnaire.

KMO value	0.817	
Bartlett spherical test	Approximate chi square *f*	2971.632
	DF	592
	*P* value	0.000

**Table 3:** CTDI-CV-modified rating standard interview.

Gauge	Subitem score	Overall score
Negative level	<15	<105
Contradiction level	15–20	105–140
Positive level	20–25	140–175
Intensity level	>25	>175

**Table 4:** Group statistics.

	Group	*N*	Mean value	Standard deviation	Standard error of mean
Achievement	Experience group	89	141.382	16.5642	1.6972
	Control group	89	137.093	20.4313	2.0986

**Table 5:** Independent sample test.

		Variance equation Levene's test		*T*-test of mean equation						
		*F*	Sig.	*T*	DF	Sig.bilateral	Mean difference	Standard error value	95% of difference confidence interval	
									Lower limit	Upper limit
Achievement	Assuming equal variance	0.408	0.519	1.260	179	0.214	3.3796	2.6982	−1.9448	8.6721
	Assume unequal variance			1.260	178.259	0.214	3.3796	2.6982	−1.9469	8.6736

**Table 6:** Pretest results of capacity.

Analysis item	Term	Sample size	Average value	Standard deviation	*T*	*P*
Seeking truth	Experience group	89	20.98	3.13	1.291	0.198
	Control group	89	20.34	3.71		
	Total	178	20.66	3.42		
Open thinking	Experience group	89	20.18	3.26	1.784	0.076
	Control group	89	19.29	3.59		
	Total	178	19.74	3.45		
Analytical reasoning	Experience group	89	21.16	3.98	0.159	0.874
	Control group	89	21.06	4.26		
	Total	178	21.11	4.12		
Systematic ability	Experience group	89	20.79	3.92	1.499	0.136
	Control group	89	19.93	4.04		
	Total	178	20.36	3.98		
Self-confidence	Experience group	89	19.71	3.71	0.423	0.673
	Control group	89	19.51	3.43		
	Total	178	19.61	3.26		
Thirst for knowledge	Experience group	89	19.48	3.27	1.412	0.160
	Control group	89	18.75	3.93		
	Total	178	19.12	3.59		
Maturity	Experience group	89	20.14	5.59	0.065	0.948
	Control group	89	20.19	5.49		
	Total	178	20.16	5.53		
Gross value	Experimental group: 142.45					
	Control group: 139.08					

**Table 7:** Group statistics.

	Group	*N*	Mean value	Standard deviation	Standard deviation of mean
Achievement	Control group	89	145.08	12.559	1.293
	Experience group	89	159.52	16.731	1.717

**Table 8:** Independent sample test.

		Variance equation Levene's test		*T*-test of mean equation						
		*F*	Sig.	*T*	DF	Sig.(bilateral)	Mean difference	Standard error value	95% of difference confidence interval	
									Lower limit	Upper limit
Achievement	Equal variance	0.036	0.845	−6.721	188	0.021	−14.442	2.149	−18.681	−10.203
	Unequal variance			−6.721	174.659	0.021	−14.442	2.149	−18.683	−10.201

**Table 9:** Differences of post-test results of thinking ability.

Group (mean soil standard deviation)				*P*
Dimension	Experimental group (*n* = 89)	Control group (*n* = 89)	*T*
Seeking truth	22.02 ± 3.09	20.87 ± 3.63	2.346	0.020
Open thinking	23.49 ± 4.56	20.89 ± 4.93	3.770	0.011
Analytical reasoning	24.96 ± 2.25	21.46 ± 3.02	9.057	0.010
Systematic ability	25.04 ± 2.12	23.14 ± 2.69	5.421	0.001
Self-confidence	21.86 ± 2.74	20.49 ± 2.69	3.475	0.003
Thirst for knowledge	21.26 ± 2.92	19.95 ± 4.64	2.340	0.021
Maturity	20.88 ± 2.70	18.27 ± 3.69	5.563	0.001

## Data Availability

The raw data supporting the conclusions of this article can be obtained from the author upon request.
